# In Silico Structural and Functional Analyses of NLRP3 Inflammasomes to Provide Insights for Treating Neurodegenerative Diseases

This article has been retracted.

**DOI:** 10.1155/2023/9819005

**Published:** 2023-01-23

**Authors:** Behram Khan Ghazi, Maria Hussain Bangash, Anam Abdul Razzaq, Madiha Kiyani, Shishay Girmay, Waleed Razzaq Chaudhary, Usman Zahid, Uzma Hussain, Huma Mujahid, Usama Parvaiz, Irfan Ahmed Buzdar, Shah Nawaz, Mohamed Farouk Elsadek

**Affiliations:** ^1^Punjab Medical College, Faisalabad, Pakistan; ^2^Basic Health Unit, 14/8R Khanewal, Pakistan; ^3^Rural Health Centre 6/G, Chishtian, Bahawalnagar, Pakistan; ^4^Department of Animal Science, College of Dryland Agriculture, Samara University, Ethiopia; ^5^Services Institute of Medical Sciences, Lahore, Pakistan; ^6^Acute & Specialty Medicine Hospital Epsom & St. Helier University Hospitals NHS Trust Medical College, Faisalabad Medical University, Pakistan; ^7^Lady Willingdon Hospital, Lahore, Pakistan; ^8^Institute of Biochemistry and Biotechnology, University of Veterinary and Animal Sciences, Lahore, Pakistan; ^9^Teaching Hospital D. G. Khan, Pakistan; ^10^Department of Anatomy, Faculty of Veterinary Science, University of Agriculture, Faisalabad, Pakistan; ^11^Department of Community Health Sciences, College of Applied Medical Sciences, King Saud University, P.O. Box 10219, Riyadh 11433, Saudi Arabia

## Abstract

Inflammasomes are cytoplasmic intracellular multiprotein complexes that control the innate immune system's activation of inflammation in response to derived chemicals. Recent advancements increased our molecular knowledge of activation of NLRP3 inflammasomes. Although several studies have been done to investigate the role of inflammasomes in innate immunity and other diseases, structural, functional, and evolutionary investigations are needed to further understand the clinical consequences of NLRP3 gene. The purpose of this study is to investigate the structural and functional impact of the NLRP3 protein by using a computational analysis to uncover putative protein sites involved in the stabilization of the protein-ligand complexes with inhibitors. This will allow for a deeper understanding of the molecular mechanism underlying these interactions. It was found that human NLRP3 gene coexpresses with PYCARD, NLRC4, CASP1, MAVS, and CTSB based on observed coexpression of homologs in other species. The NACHT, LRR, and PYD domain-containing protein 3 is a key player in innate immunity and inflammation as the sensor subunit of the NLRP3 inflammasome. The inflammasome polymeric complex, consisting of NLRP3, PYCARD, and CASP1, is formed in response to pathogens and other damage-associated signals (and possibly CASP4 and CASP5). Comprehensive structural and functional analyses of NLRP3 inflammasome components offer a fresh approach to the development of new treatments for a wide variety of human disorders.

## 1. Introduction

Inflammasomes are multiprotein complexes that have the inherent capacity to trigger an innate immune reaction upon the detection of a molecular pattern (also known as a PAMP) or a damage-associated molecular pattern (also known as a DAMP) [1]. Pattern recognition receptors (PRRs) are specialised structures that can be found in the cytoplasm (for example, RIG-I-like receptors: RLRs), on the cell surface (for example, Toll-like receptors: TLRs), or in endosomal compartments (for example, RIG-I-like receptors: RLRs) [2]. These molecular patterns are recognized by these PRRs. When these PRRs are activated, downstream signalling pathways are triggered, which ultimately result in the release of cytokines that promote inflammation [3]. It is necessary for certain of these cytokines to undergo further processing before they can perform their intended role. This procedure occurs after cytokines have been released into the bloodstream [3, 4]. PRRs, which lack melanoma 2-like receptors (ALRs, AIM2-like receptors) and possess nucleotide-binding oligomerization domain- (NOD-) like receptors (NLRs), are the essential components of the inflammasome complex [5]. PRRs contain nucleotide-binding oligomerization domain- (NOD-) like receptors (NLRs). Among the many inflammasomes identified to date are the NLR family member NLRP3, as well as NLRP1, AIM2, and NLRC4. NLRP3 is an intracellular sensor that is a part of the inflammasomes [6]. It is the NLRP family member that recognizes the widest array of PAMPs (pathogen-associated molecular patterns) and DAMPs (danger-associated molecular patterns). The three domains that make up NLRP3 are an ATPase-active NACHT domain, an LRR domain that causes autorepression by folding back onto the NACHT domain, and an amino-terminal pyrin domain (PYD) that binds to ASC [7]. Research has focused on the ATPase activity of the NACHT domain in particular as a possible therapeutic target for NLRP3-related diseases [8]. NLRP3 is composed of three distinct structural domains: an N-terminal pyrin domain, a central adenosine triphosphates (ATPase) domain referred to as NACHT, and a C-terminal leucine-rich repeat (LRR) domain. It has been reported that the chemical MCC950, which is based on a sulfonylurea structure, is an effective inhibitor of NLRP3 [9]. MCC950 was shown in recent research [10] to suppress NLRP3 in a manner that does not involve covalent bonding. It seems to bind at the area proximal to the Walker B motif [11, 12], which is located inside the NACHT domain, and this has an effect on the activity of the protein. The involvement of NLRP3 has also been identified to contribute to the pathophysiology of disorders of the central nervous system, such as Alzheimer's disease [13] and Parkinson's disease [14]. Intestinal cancer and autoimmune inflammatory illnesses including keratitis and conjunctivitis have been linked to abnormal activation of the NLRP3 inflammasome [15, 16]. As a result, the finding of pharmacological inhibitors that target NLRP3 inflammasome components offers a fresh approach to the development of new treatments for a wide variety of human disorders. Furthermore, genetic polymorphisms and mutations in NLR-coding genes and inflammasome sensor proteins have been linked to a wide range of autoimmune disorders [4]. Because of this link to numerous illnesses, therapies that target inflammasome activity have been developed. The biological system's complexity has cleared the way for cutting-edge machine learning (ML) techniques in the identification and development of pharmaceuticals with improved therapeutic effectiveness [17]. However, the process of creating novel NLRP3 modulators is made more difficult since there is a paucity of structural knowledge regarding the oligo-protein, and the molecular mechanism of current inhibitors is not completely understood. In the current study, we constructed a homology model of the protein, and we utilised it in a computational process to uncover probable protein binding sites that are engaged in the stabilization of the protein-ligand complex with the inhibitors, with the goal of gaining a deeper comprehension of the molecular process behind their interaction.

## 2. Materials and Methods

### 2.1. Sequence Retrieval

We searched for the human NLRP3 nucleotide and amino acid sequences in the online databases of Ensembl (ENSG00000162711) [18] and the National Centre for Biotechnology Information (NCBI) (https://www.ncbi.nlm.nih.gov) [19]. Ensembl is a part of the National Institutes of Health. We were able to get the crystal structure of the protein by consulting the public database of the Protein Data Bank (PDB) at http://www.rcsb.org [20].

### 2.2. Protein Structure Prediction

The human NLRP3 protein sequence was retrieved in FASTA format from UniProt (accession no. Q96P20) and used as a query for BLAST against a nonredundant protein database at http://blast.ncbi.nlm.nih.gov/Blast.cgi. The retrieved protein sequences were aligned using the multiple sequence alignment technique Clustal Omega (version 1.2.4) [21]. The PSI-BLAST server (http://blast.ncbi.nlm.nih.gov/Blast.cgi) was queried with the same sequence as a query against the PDB to identify structural homologs [22]. The alignment of the query sequence with the template sequence was accomplished with the help of PRALINE (http://www.ibi.vu.nl/programs/pralinewww/) [23]. The UCSF-Chimera 1.10.1 software was utilised to see the 3D-modelled structure of proteins. UCSF Chimera is a tool for the interactive viewing and study of structural features and associated data, including the protein's density. Protein structure analysis (ProSA), a method for identifying flaws in theoretical and empirical protein structures, was one of the tools we employed in our investigation to validate protein structure [24]. The ProSA web software language is designed to validate atomic structure coordinates based on predictions, and the results are scored according to *z* score values. ProtParam [25] was used to calculate theoretical Pis, extinction coefficients, aliphatic and instability indices, and GRAVY values for each of these variables.

### 2.3. Analysis of NLRP3 Protein Ligands and Domain

Understanding the functional component of a protein's structural characteristic is important for proteomics; as a result, multiple bioinformatics methods were used to predict the NLRP3 protein's ligand, ligand-binding sites, and domains. In addition, the protein ligands were grouped according to how similarly they served a purpose. RaptorX, a template-based, reliable 3D modelling online tool, predicted the protein structures' ligand-binding residues [26]. RaptorX is renowned for producing structural modelling output of the highest calibre for several targets utilising a single remote template. I-TASSER was used to identify binding site number with the locations, and several additional programmes were utilised to cross-check and confirm the dependability and correctness of the anticipated outcome, including COACH server [27, 28]. By leveraging the BioLiP posttranslational modification database to identify ligand-binding sites, COACH is a meta-server strategy for identifying ligand-binding targets. It compares two approaches, TM-SITE [29] and S-SITE [30]. We utilised the ligand-binding prediction tools available on the FTSite website [31] in order to gain an understanding of the ligand-binding surface on the nonbound portion of the freely existing protein structure. According to the reports, its accuracy is on par with the outcome of the trial [31]. The FTSite prediction concept is based on fragments of data gleaned from the experiment rather than being template- or evolutionary-based [32, 33].

The LPIcom web server [34] accessible at http://crdd.osdd.net/raghava/lpicom performed ligand module clustering to better comprehend the interaction between the ligands and amino acids of the target protein. Additionally, utilising the LPIcom web server, residues, preferred interactions, and binding motifs for a specific ligand were predicted. All target proteins' domains were looked up in NLRP3 using InterProScan [35] and the protein domain database [19]. The photos were then precisely and succinctly visualised using DOG 2 software [36].

### 2.4. Protein Interactions and Coexpression Analysis

Evaluation of the functional connections that take place within the cell must first and foremost focus on the interactions that take place between different proteins. In order to identify NLRP3 protein interactions with other proteins, the Search Tool for Retrieving Interacting Genes/Proteins (STRING) database (https://string-db.org) was used [37]. Using its database of 24,584,628 proteins from 5090 species, the database generated protein-protein interactions via direct or indirect links between the NLRP3 protein and other proteins. NLRP3 as a gene and Homo sapiens as an organism were entered as the input query for this investigation. Both the functional and the physical interactions between proteins are taken into account by the STRING software tool [38]. The software approach was built to capture protein-protein interaction based on the previous research, empirical output, data mining, and cooccurrence [39].

### 2.5. Predicting Consensus Sequence Alignment and Secondary Structure

A free open-access application called ENDscript 2 was used to display different biochemical and structural modifications in order to better understand how NLRP3's structure aligns [40]. The online tool was created such that it can distinguish between primary and quaternary structures, which range in complexity from simple to complicated. Additionally, it makes use of the PDB input format and divides its results into a number of categories that may be seen in a variety of structural interface tools. Additionally, the secondary structure of the protein was estimated using PSIPRED version 3.3 [41], an online programme that integrates protein sequence and computational modelling onto a single platform. Initially, PSI-BLAST is run on input data pertaining to protein sequences.

### 2.6. Evolutionary Conservation Analysis

Utilising the ConSurf web server (http://consurf.tau.ac.il/), an investigation on the degree to which the individual amino acids that make up the NLRP3 protein are evolutionary conserved was carried out [42]. For the purpose of resolving evolutionary conservation and the categorization of potential structural as well as functional residues in the NLRP3 protein, the ConSurf algorithm makes use of a technique that takes an empirical Bayesian approach. The final score may be broken down as follows: variable conservation between 1 and 4, moderate conservation between 5 and 6, and well conserved between 7 and 9 [32].

### 2.7. Transcriptomic Analysis

In order to explore the NLRP3 gene expression, the Genotype-Tissue Expression (GTEx) archive (dbGaP, accession number phs000424.v8. p2) was utilised [43]. This archive contains gene-level association data that demonstrates the screening and regulating effect of gene expression levels on phenotypes. In order to search a bulk tissue expression panel, we made use of the phrase “NLRP3” in conjunction with the gene data (ENSG00000162711.16). This project's goal is to create a comprehensive online resource that can be used to gain a deeper understanding of the expression and regulation of genes that are specific to various tissues. Nearly one thousand people had healthy tissue samples collected from 54 different locations on their bodies so that molecular analyses could be carried out on them [43].

## 3. Results

### 3.1. Gene Cooccurrence and Evolutionary History

We identified probable split genes inside the multiple alignment by looking for occasions where suspected split gene sequences did not overlap. A representative protein was utilised for each protein-coding gene in Ensembl. Scores obtained from BLAST are input into hcluster so that it may organise the sequences into gene families. Following the alignment of the proteins using either MCoffee or MAFFT, a phylogenetic tree was constructed using TreeBeST. In conclusion, orthologues and paralogues are deduced from the tree using the information provided. In order to construct the phylogenetic tree, alignments from both Infernal and PRANK were utilised, and then, the tree was combined with TreeBeST to form the final model. At last, orthologues and paralogues were deduced from the tree using the information provided. Every protein that can be found in Ensembl and every metazoan protein that can be found in UniProt are utilised. Scores from BLAST are input into MCL, which then organises the sequences according to their degree of similarity. The MAFFT algorithm was used to align the proteins. Gene trees help with the evolutionary history of gene families, evolving from a common ancestor. For inferring orthologues and paralogues, duplication and speciation events are distinguished, reconciling the gene tree against the species trees. As a simple case of unique orthologous genes concern, reciprocal best approaches show a clear concordance. Still, concerning more complex one-to-many and many-to-many relations, the gene tree pipeline is considered the best. This approach can significantly raise the orthologues number of hominines to mammal and has even more extreme effects on the orthologous gene in mammal predictions. Furthermore, it aids in exploring the time duplication events that result in paralogues by ascertaining the most recent common ancestor (i.e., taxonomy level) for a given internal node of the tree (Figure 1).

The final tree, also known as the consensus tree, is built by merging the five individual trees using an algorithm designed specifically for tree merging. These allow TreeBeST to leverage DNA-based trees and protein-based trees for closely connected sections of trees and distant connections, respectively, and that a set of algorithms may overtake others in particular cases. In addition, this enables TreeBeST to utilise the fact that protein-based trees are more accurate than DNA-based trees. An individual consensus tree is produced as a result of the simultaneous consolidation of five input trees by the method. The consensus topology has clades included from all of the input trees, which helps to limit the amount of duplicates and losses that are inferred and achieves the maximum bootstrap percentage. The HKY model is used in phyml to make estimates of the branch lengths that are based on the DNA alignment of the final consensus tree.

### 3.2. Protein Domain Analysis and Structure Prediction

The programme InterPro was used to figure out the structural components of the NLRP3 protein as well as the locations of variations. Proteins are categorized into their respective protein families and then subjected to a functional analysis by InterPro. It provides an additional estimation of the look of active websites and domains. Therefore, the NLRP3 protein is a member of the NLRP family that identifies the most diverse set of PAMPs and DAMPs. These acronyms stand for pathogen-associated molecular patterns and danger-associated molecular patterns, respectively (DAMPs). The NACHT domain and the LRR domain were discovered to be present (Figure 2). In addition, the secondary structure of the NLRP3 protein has been determined by using PSIRED, and it has been shown that the secondary structure has a heterogeneous distribution of coils, helices, and strands (Figure 3). RaptorX, a web server used to evaluate 3D protein structure modelling, was used to predict the secondary structure of the human NLRP3 protein. The beta helix is represented by a blue arrow, the coil by a yellow arrow, and the alpha helix by a red arrow. Residues are shown in a conformation that flips out of the active site in structure three subunits (Figure 4), but this conformation is unusual in that it is oriented towards the active site.

### 3.3. Protein-Ligand Interactions

The protein-ligand-binding site residues predicted by PDB sum and visualised by both LIGPLOT and PLIP are provided for NLRP3 protein (Figure 5). For each binding site, an interaction diagram along with the associated interaction data is presented. Two ligands ADP and 8GI interacting with various binding locations have been identified in NLRP3 protein. The residues of the amino acids A227, I230, G231, L232, T 233, I234, and H522 were involved in bonding interactions with ADP, while G229, P373, T381, and L413 were nonbonding interactions with ADP. Compound ADP displayed strong binding energy, which might be because the methyl group was substituted. It was found that the hydrogen bonding produced by compound ADP was of moderate strength. A227, A351, I411, T443, M408, P575, L628, and T632 were the amino acid residues engaged in nonbonding interactions with 8GI, while A228, A578, and G629 were involved in bonding interactions with 8GI (Figure 5).

### 3.4. Physicochemical and Conservation Analysis

Several fundamental biological processes rely on the positional behavior of amino acids, whether located in catalytic sites or elsewhere, as is required for protein interactions. As a consequence of this, certain amino acids end up being more recognizable and stable than the many residues that make up a specific protein sequence. Amino acid variations that are positioned at locations that have been evolutionarily conserved are expected to give rise to more damaging mutations than amino acid variations found at places with less conversed positions. Applying the ConSurf algorithm to the amino acids of the human NLRP3 protein and looking at it from an evolutionary perspective allowed for the determination of the rate of conservation, which was relevant to the more sophisticated study of the likely impacts of the high-risk SNPs.

Consequently, amino acid locations that are affected by high-risk SNPs are a plausible scenario; despite this, ConSurf also verifies other residues that might possibly hold significant practical importance. As a consequence of this, mutations with a higher score for evolutionary conservation are considered to carry a greater potential for generating illness. Estimating a protein's structural or functional foundation can be aided by looking at the conserved regions closer to its surface or deeper into its core. According to the results of a ConSurf study, the majority of the residues in the NACHT domain have scores ranging from 7 to 9, but the LRR domain has a prediction of fewer conserved residues, with an average conservation value of 6 (Figure 6). Interestingly, ConSurf recognized the majority of the conserved residues with greater conservation as being structurally or functionally significant residues. The structural constancy of a protein involves interresidue communications. These interactions' energetic influence can be estimated by low-resolution force fields achieved from recognized structures based on amino acid composition and frequencies. We analyzed human and mouse NLRP3 protein sequences using NPS@: Network Protein Sequence Analysis online server (https://npsa-prabi.ibcp.fr/cgi-bin/npsa_automat.pl?page=/NPSA/npsa_server.html). We found that NLRP3 protein comprised of 22 amino acids, the most abundant residue is alanine, which is 11.05% and 11.76% of total protein, and the other large residue is glutamic acid, which is 10.06% and 9.01% of the protein (Table 1).

A ProtParam tool was used to calculate the anticipated structure of the targeted proteins' physicochemical properties in order to confirm the reliability of the anticipated structure even further. Following these steps allowed for the calculation of the values for several physicochemical characteristics, such as the theoretical pI, estimated half-life, aliphatic index, and extinction coefficients. When calculating the PI score of the target proteins, the principle of pK values was taken into consideration. The PI scores for human NLRP3 were then obtained, and the results showed that they were comparable to the ranges of PI values reported for proteins in earlier research [45], indicating that the currently predicted value is within the standard range (Table 1). The GRAVY values, which are a measurement of the hydropathy features of the residues of the specific proteins [40], have been determined. As shown in Table 1, it is anticipated that the NLRP3 will have a negative value, which will indicate that it is more hydrophobic.

### 3.5. Gene Expression across Tissues of NLRP3 Gene

The expression quantitative trait locus (eQTL) browser is a fundamental component of the GTEx database. This database stores and makes accessible the results of a national study that sought to establish a connection between genetic variants and high-throughput molecular-level expression phenotypes. A significant number of genes have been shown to be associated with a number of tissues. The NLRP3 inflammasome has been implicated in a wide variety of physiological and pathological processes, including inflammation, apoptosis, and necrosis. The expression of the NLRP3 inflammasome was much higher in the cell bodies and axons of the prefrontal cortex, hippocampus, and peripheral blood monocytes (PBMCs) (Figure 7). The investigation of changes in gene expression at the exon level can be demanding but ultimately worthwhile. Even the more advanced algorithms have limits when it comes to expressing the transcript levels in absolute terms. Exon level information concerning the kind and quantity of transcripts has previously been found to be more illuminating [46]. With the understanding that more than 90% of all genes are subject to alternative splicing, which results in the production of several transcripts for a single gene, the potential of exon level data is now more fully exploited than ever [47]. The gene-centric strategy to carrying out integrated analysis with the help of aCGH and exon array data has produced more confirmed results, but it does not make full use of the possibilities offered by whole genome arrays [48]. However, when we averaged across all (significant) genes using different metrics for enrichment, tissues that were projected to be more enriched for diseases and currently understood biology did not always do so. There are some interesting relationships that point to several tissues being involved. It is possible that this is due to how sensitively different contexts affect different regulatory mechanisms. We determined the number of splicing events (exons, splice junctions, and transcripts) by measuring the percentage of spliced-in exons. Clustering the samples according to their PSI scores also broadly, but not as clearly, recapitulates the kind of tissue. The major outgroup, which can be seen in figure and is comprised of two groups, is comprised of samples taken from the brain rather than the blood. A smaller group (cluster 2), which is dominated by the remaining subregions, clusters nearer to samples from the remaining tissues than a larger group (from the cerebellum and cortex) that form an independent sub cluster (cluster 1) (Figure 8).

### 3.6. Prediction of FT Site

Accurately pinpointing protein-ligand-binding sites has far-reaching implications for many fields of biology, including but not limited to drug discovery, protein modelling, and engineering. To determine if the NLRP3 protein has an epitope or a protein binding area, we utilised the FT site server available at http://ftsite.bu.edu/ to predict binding sites in the NLRP3 protein. Using an energy-based procedure, the FT site server can correctly predict ligand-binding sites 94% of the time in experiments. Three ligand-binding sites were found for our target protein by using the FT site server, and the ligand-binding sites were identified using the native NLRP3 protein (Figure 9).

### 3.7. Protein-Protein Interaction and Coexpression Analysis

The STRING performed a coexpression analysis database that showed coexpression scores based on RNA expression patterns and protein coregulation provided by Proteome HD. For human NLRP3, the coexpression score was 0.179. It was found that human NLRP3 gene coexpresses with PYCARD, NLRC4, CASP1, MAVS, and CTSB based on observed coexpression of homologs in other species. The NACHT, LRR, and PYD domain-containing protein 3 is a key player in innate immunity and inflammation as the sensor subunit of the NLRP3 inflammasome. The inflammasome polymeric complex, consisting of NLRP3, PYCARD, and CASP1, is formed in response to pathogens and other damage-associated signals (and possibly CASP4 and CASP5). The process of recruiting proCASP1 to the inflammasome speeds up its activation, which in turn speeds up the maturation and secretion of IL1B and IL18 in the extracellular milieu, which are both catalyzed by CASP1. It is also necessary for the activation of the NLRP3 inflammasome in order for HMGB1 to be secreted (Figure 10).

## 4. Discussion

The NLRP3 inflammasome has been activated by a variety of stimuli, but the precise mechanism is still unknown and is the subject of ongoing research. Additionally, research has shown that posttranslational changes play a crucial role in the activation of NLRP3 [49, 50]. However, it has been discovered that NLRP3 inflammasome inactivation is induced by ubiquitination and posttranslational changes during the priming step [51], whereas its activation is induced by dephosphorylation and deubiquitination [52]. Additionally, NLRP3 inflammasome deactivation depends on protein kinase A-associated NLRP3 phosphorylation on position Ser291 [4]. Furthermore, recent research revealed the role of microRNAs in the control of the NLRP3 inflammasome.

Using homology-modelling methods, we began to use in silico research by performing a 3D structural modelling for human NLRP3 [53]. This modelling was done using a computer simulation. The human NLRP3 three-dimensional models that were predicted have displayed a variety of colours, features, and conformations in their structures (Figure 2). Validations of the three-dimensional models of two proteins were performed once the modelling of their structures in three dimensions was completed. We determined that the NLRP3 proteins in all species have amino acid sequences that are conserved around the ligand-binding region. Additionally, the three-dimensional structures of NLRP3 are remarkably comparable to one another. This was revealed by studying the essential active sites of the NLRP3 protein sequences of diverse species [54]. It was also shown that the spatial structure of both human and mouse NLRP3 contain a common receptor protein that has a serine/threonine kinase activation site. This finding suggests that the activities of the NLRP3 genes in human and mouse could be comparable. Bioinformatics technologies can be used to bridge the gap between the amount of protein sequences and their 3D structure. Computational tools are being utilised more and more frequently to narrow the search in sequence space, which increases the effectiveness of laboratory evolution [55]. Adiyaman and McGuffin [56] acknowledge that in silico protein modelling is more cost-effective and faster than traditional methods of protein characterization. Protein structure and function can be studied both quantitatively and qualitatively using in silico methods such as protein structure analysis [57]. To better understand proteins' structure and function, in silico research of proteins has made significant contributions to computational biology in the last few years [58]. The evolutionary, structural, and functional analyses of the human NLRP3 inflammasome have been taken into consideration in the current study [59]. In the current investigation, the cooccurrence of genes was analyzed, and an evolutionary tree was developed to identify the history of families. According to the findings, NLRP3 proteins from various species were discovered to be remarkably comparable in humans and other mammals; hence, it is hypothesized that they are descended from a single ancestor (Figure 1). These results are consistent with a prior study, which indicated that the NLRP3 gene sequence was determined to be highly conserved throughout vertebrate evolution. However, within that species, there were numerous copies of that gene, and those copies exhibited a significant presence among paralogues. Similar to this, another study found that the best way to understand the diversity and function of the NLRP3 genes is by building a phylogenetic tree [60].

In this study, the ProtParam server was used to assess the primary structure of NLRP3 and other physicochemical parameters inferred from protein sequences in order to predict gene structure and function. Theoretical pI (isoelectric point), molecular weight, atomic composition, amino acid composition, predicted half-life, extinction coefficient, instability index, high hydropathicity, and aliphatic index are some of the properties that were measured. The NACHT domain and the LRR domain were discovered to be present (Figure 2). In addition, the secondary structure of the NLRP3 protein has been determined by using PSIRED, and it has been shown that the secondary structure has a heterogeneous distribution of coils, helices, and strands (Figure 3). RaptorX, a web server used to evaluate 3D protein structure modelling, was used to predict the secondary structure of the human NLRP3 protein. According to the findings, the majority of the NLRP3 was organised as an alpha helix or a random coil. Human NLRP3 has been used as a sample of other organisms by the Phyre2 server to predict their tertiary structures. On the other hand, it was recently discovered that MCC950 binds to the NACHT domain [58] and that this binding takes place at a region that is most likely close to the Walker B motifs and these are the protein sequence patterns that have extremely conserved three-dimensional structures. In order to accomplish this goal, we conceived of three distinct techniques, each of which would use algorithms based on either docking, grids, or geometry, in that order. FTMap [61] was chosen for the examination of the protein structure's suitability as a therapeutic target. To map the protein, the computational mapping service known as FTMap employs a set of probes consisting of 16 tiny molecules that vary in terms of their size, shape, and polarity [62]. FTMap does this by clustering each probe type according to the protein region, which identifies possible hot sites for protein binding. Estimating a protein's structural or functional foundation can be aided by looking at the conserved regions closer to its surface or deeper into its core. According to the results of a ConSurf study, the majority of the residues in the NACHT domain have scores ranging from 7 to 9, but the LRR domain has a prediction of fewer conserved residues, with an average conservation value of 6 (Figure 6). Interestingly, ConSurf recognized the majority of the conserved residues with greater conservation as being structurally or functionally significant residues. The structural constancy of a protein involves interresidue communications. The NLRP3 inflammasome has been implicated in a wide variety of physiological and pathological processes, including inflammation, apoptosis, and necrosis [63]. The expression of the NLRP3 inflammasome was much higher in the cell bodies and axons of the prefrontal cortex, hippocampus, and peripheral blood monocytes (PBMCs) (Figure 7). The investigation of changes in gene expression at the exon level can be demanding but ultimately worthwhile. Even the more advanced algorithms have limits when it comes to expressing the transcript levels in absolute terms. Exon level information concerning the kind and quantity of transcripts has previously been found to be more illuminating [64].

## 5. Conclusion

Despite the pathway's intricacy, there has been some advancement in the creation of treatments that focus on the NLRP3 inflammasome and the pathways it is connected to. However, additional knowledge is required to completely define the pathways that will expand our understanding of how to discover exact medication targets and which ones may result in more effective treatments. In this context, the investigation of cutting-edge technologies such as artificial intelligence and machine learning is building the groundwork for the creation of medicines that are more effective. Because of this, conducting an in silico investigation of the physicochemical properties of a protein is extremely crucial if one want to obtain a theoretical overview of an enzyme. This paper gives the very first structural analysis of human NLRP3 that has been disclosed. Nevertheless, additional clarity is required regarding the regulatory systems and the role that they play in the progression of the disease. The recent finding of the NLRP3 inflammasome has presented researchers with a fresh window of opportunity to investigate the pathophysiology of disorders that are associated with inflammation. In-depth study of the NLRP3 inflammasome, which controls IL-18 and IL-1b, will offer a fresh approach to the management and prevention of inflammatory illnesses. By comparing the results of genomes and transcriptional investigations, we were able to obtain a greater understanding of the NLRP3 gene.

## Figures and Tables

**Figure 1:** Gene tree displaying genes that have been divided. GeneTree database entry for the NLRP3 gene in version 80 of the Ensembl database. The nodes in the tree that are coloured blue signify instances of speciation, whereas the nodes that are coloured light brown represent gene splits. The distinct species clades are shown by the varied colours of the backdrop. Some of the nodes in the tree have been compressed into grey triangles, which display a synopsis of the subtree they belong to. The right side of the picture provides an overview of the alignment, with the gaps in the protein alignments shown by white patches. The three instances of gene splitting that occurred in this family are shown by the three light brown rectangles. The alignment summary for these genes demonstrates quite clearly how the genes were separated into their respective parts.

**Figure 2:** Molecular structure of NLRP3 conserved domain analysis. The human NLRP3 crystal structure was utilised as a reference, and using the Phyre tool (http://www.sbg.bio.ic.ac.uk/phyre2/html), all chains in the protein were plotted onto the crystal structure.

**Figure 3:** A topology diagram depicting the NLRP3 protein. NLRP3 secondary structure “wiring diagrams” that show alpha helices, beta sheets, and other motifs like alpha and beta turns and the amino acid strings that correspond to those motifs. The protein sequence for human NLRP3 is depicted in the figure below, along with the secondary structure elements that have been ascribed to it. Human NLRP3 topology diagram (PDB: 7pzc). The PDBSUM server was utilised in the creation of the figure [44].

**Figure 4:** Secondary protein structures of NLRP3. Letters are used to identify the conserved residues, and the tertiary structure's representation of helices is colour coded. Beta sheets, coils, and the alpha helix are all shown in red arrows in this protein structure diagram. Human NLRP3 can be seen in the upper panel.

**Figure 5:** Predicted ligand-binding site of human NLRP3 protein. Hydrogen bonds are denoted by dashed lines that run between the atoms that are involved, whereas hydrophobic interactions are depicted as an arc with spokes that radiate towards the binding atoms that they contact. The atoms that have made contact are represented by spokes that radiate backward.

**Figure 6:** Conservation analyses of PRKAG3 protein of Yak. Amino acid conservation was predicted using a scale from 1 to 9 based on the conservation value of each individual amino acid; values of 1-4 indicate low conservation, 5-7 suggest moderate conservation, and 8-9 indicate high conservation.

**Figure 7:** Tissue expression profile of human NLRP3 gene has their own unique expression. The expression data of the genes that were suggested across a variety of human tissues, courtesy of the GTEx collaboration [46].

**Figure 8:** Clustering of gene expression and exon splicing profiles of NLRP3 gene.

**Figure 9:** The human NLRP3 protein's predicted FT binding site. Zoom in on ligand-binding sites 1 (pink-coloured mesh), ligand-binding sites 2 (green-coloured mesh), and ligand-binding site 3 (blue-coloured mesh) in FT site prediction, where pink, green, and blue colours, respectively, indicate the first, second, and third binding sites in protein chains (a–i) (blue-coloured mesh).

**Figure 10:** Analysis of the protein-protein interactions that occur between NLRP3 inflammasome and other proteins. The distance between interacting proteins can be determined, in part, by the length of the link between them. Nodes that do not represent known proteins are highlighted in red, whereas nodes that do represent known proteins are shown in full. The connections between the proteins are represented by the black lines. Scores for coexpression that are offered by Proteome HD and are derived from RNA expression patterns and protein coregulation. An examination of the network formed by human NLRP3 and other species.

**Table 1:** Physicochemical properties of human NLRP3 proteins.

Parameters	Values
Number of amino acids	1034
Molecular weight	117913.21
Theoretical pI	6.17
Extinction coefficients	119980
Estimated half-life	30 hours
Instability index	45.36
Aliphatic index	93.06
Hydropathicity (GRAVY)	-0.201

## Data Availability

All materials and data will be available to the readers without undue qualifications in material transfer agreements.
